# Long-Term Stability of Hydromorphone in Human Plasma Frozen at −20°C for Three Years Quantified by LC-MS/MS

**DOI:** 10.1155/2022/3645048

**Published:** 2022-06-28

**Authors:** Andreas Wehrfritz, Stefanie Schmidt, Harald Ihmsen, Jürgen Schüttler, Christian Jeleazcov

**Affiliations:** Department of Anesthesiology, University Hospital Erlangen, Friedrich-Alexander-University of Erlangen-Nürnberg (FAU), Krankenhausstrasse 12, 91054 Erlangen, Germany

## Abstract

The long-term stability of drugs under normal laboratory storage conditions (−20°C) for years is important for research purposes, clinical re-evaluation, and also for forensic toxicology. To evaluate the stability of the analgesic opioid hydromorphone, 44 human frozen plasma samples of a former clinical trial were reanalyzed after at least three years. Blood samples were disposed using solid-phase extraction with an additional substitution of stable isotope labelled hydromorphone as an internal standard. Hydromorphone concentrations were determined by ultra-performance liquid chromatography (UPLC) with gradient elution, followed by tandem mass spectrometry with electrospray ionization. Calibration curves demonstrated linearity of the assay in the concentration range of 0.3–20 ng/mL hydromorphone. The limit of detection of the hydromorphone plasma concentration was 0.001 ng/mL, and the lower limit of quantification was 0.3 ng/mL. Intra- and interassay errors did not exceed 16%. The percentage deviation of the measured hydromorphone plasma concentrations between the reanalysis and the first analysis was −1.07% ± 14.8% (mean ± SD). These results demonstrate that hydromorphone concentration in human plasma was stable when the samples were frozen at −20°C over three years. This finding is of value for re-evaluations or delayed analyses for research purposes and in pharmacokinetic studies, such as in forensic medicine.

## 1. Introduction

Hydromorphone (4,5alpha-epoxy-3-hydroxy-17-methylmorphinan-6-one) is an analgesic opioid with sevenfold stronger analgesic potency than morphine [1], which is commonly used for the relief of strong acute and chronic pain [2]. All opioid analgesics are accompanied by misuse even if hydromorphone is not the first-line opioid for abuse and addiction [3]. High-potency opioids such as hydromorphone might independently influence the risk of suicide as well [4]. On the other hand, there are efforts to expand the access to hydromorphone as an opioid substitution option in some countries [5].

The analysis of blood samples taken some time ago can be relevant not only in forensics but also in pharmacology, for example, for external validation of pharmacokinetic models using existing blood samples. The effect of storage on analyte concentrations is also relevant from a laboratory point of view, as incorrect storage is one of those preanalytical problems, which can account for 60–70% of all errors occurring in the entire testing process [6]. Therefore, the long-term stability of an analyte is a question of importance. Substances that have been studied for long-term storage include morphine, codeine, and 6-acetylmorphine [7], as well as benzodiazepines and other opioids [8]. Recently, Truver and Swortwood-Gates demonstrated the long-term stability of novel synthetic opioids over a 36-week period in blood [9].

The guidelines for the bioanalytical method validation of the Food and Drug Administration (FDA) state that long-term stability should be assessed over a period of time equal to or exceeding the time between the date of first sample collection and the date of last sample analysis [10]. In a clinical phase III study, this time period can last up to one year, as it was the case in a study on hydromorphone which we had conducted previously [11]. Therefore, the minimum time period for the assessment of the long-term stability of hydromorphone should be one year. On the other hand, investigations to further develop, refine, or validate a pharmacokinetic/pharmacodynamic model are typically conducted up to 5 years after a model is developed, as it was the case for a validation study on hydromorphone which we conducted in 2014 and 2015 [12], while the pharmacokinetic model had been developed in a study in 2011 and 2012 [11]. Therefore, we considered a time period of about 3 years as reasonable for the assessment of the long-term stability of hydromorphone. Surprisingly, the stability of hydromorphone concentrations after long-term storage has not been studied to date, although it has a higher analgesic potency than morphine. Hildebrand et al. reported that the concentration of hydromorphone in infusion systems was stable over a medium-term period of four months [13]. Another study found that hydromorphone in 0.9% sodium chloride was also stable in a medium-term period for at least 50 days when stored at room temperature in polypropylene syringes [14]. Other validated methods quantified the medium-term stability of hydromorphone for a maximum of ten days [15, 16]. Saari et al. validated the stability of hydromorphone over 3 months using a specific and sensitive method for liquid chromatography-tandem mass spectrometry (LC-MS/MS) which was developed to quantify the concentration of total and unbound hydromorphone in patients undergoing cardiac surgery [17].

To our knowledge, the stability of hydromorphone dissolved in human plasma for a longer period of several years has not yet been reported. Therefore, it was the aim of the present investigation to analyze the long-term hydromorphone stability in human plasma frozen at −20°C for at least three years. Based on the analytical method by Saari et al., samples were reanalyzed by a slightly modified and enhanced method which we had previously developed to determine morphine and morphine-6-glucuronide [18].

## 2. Materials and Methods

### 2.1. Samples

We reanalyzed 44 plasma samples of three patients who had participated in a clinical study on postoperative pain therapy with hydromorphone after cardiac surgery, which was performed at the Department of Anesthesiology of the University Hospital of Friedrich-Alexander-University, Erlangen, Germany, in 2016 (ClinicalTrials.gov identifier: NCT02483221). The trial was performed in accordance with Good Clinical Practice (GCP) and the Declaration of Helsinki. Ethical approval was provided by the Ethics Committee of the University of Erlangen. These 44 plasma samples had been frozen at −20°C for at least three years.

### 2.2. Drugs and Chemicals

Hydromorphone (1 mg/mL in methanol) and internal standard (IS) hydromorphone-D3 were purchased from LGC Standards (Wesel, Germany). Water for the mobile phase (ROTISOLV®), acetonitrile, methanol, formic acid, and ammonia (30%) were purchased from Roth (Karlsruhe, Germany); all chemicals and solvents were high-performance liquid-chromatography (HPLC) grade. Deionized water for the solid-phase extraction was prepared with a Simplicity® system from Millipore (Schwalbach, Germany). Lyophilized drug-free human serum was obtained from Bio-Rad Laboratories (Feldkirchen, Germany), and each vial was reconstituted with 10 mL of LC-MS/MS grade water for use.

### 2.3. Standard Solution and Calibration Standards

Two stock solutions of hydromorphone and hydromorphone-D3 were prepared by dissolving the standards with methanol in a concentration of 20 ng/mL and stored at −20°C. Standard working solutions for calibration, validation, and quality control samples were obtained by further dilution of the stock solution with methanol. Calibration samples with concentrations of 20, 10, 5.0, 2.5, 1.25, 0.63, and 0.31 ng/mL were used for the determination of the total hydromorphone concentration. Quality control (QC) samples were used in concentrations of 20, 2.5, and 0.31 ng/mL. All analytical samples were prepared to drug-free plasma and blank study plasma samples (zero samples) by adding 50 *μ*l hydromorphone standards to 450 *μ*l drug-free plasma. All standards were prepared for the LC-MS/MS analysis according to the plasma sample preparation.

### 2.4. Sample Preparation

Before further preparation, the three years stored, long-time frozen (−20°C) plasma samples were thawed and centrifuged for 5 min at 2000 × *g*. For extraction, OASIS HLB solid-phase extraction cartridges (Waters, Eschborn, Germany), conditioned with 2 mL of methanol, were supplied with aliquots of 450 *μ*L plasma and 50 *μ*L of 20 ng/mL hydromorphone-D3 as the internal standard. Cartridges were rinsed twice with 1 mL water and were further centrifuged for 1 min at 2000 × *g* to descale the residual water. Analytes were first eluted under a slight vacuum with 0.9 mL acetonitrile, containing 5% ammonia, and subsequently evaporated to dryness under nitrogen. Finally, analytes were reconstituted with 200 *μ*L water and 0.1% formic acid to get a mobile phase compatible with the electrospray ionization interface (ESI). An aliquot of 5 *μ*L of the extracted sample was injected in the UPLC system.

### 2.5. Equipment

Waters Alliance Separation Module 2695 for chromatographic separation and a Quattro micro tandem mass spectrometer (Waters, Eschborn, Germany) were used for analyses of the extracted substances. This system was upgraded and modified by Fischer analytics (Bingen, Germany) to allow UPLC-like pressures of more than 400 bars. For chromatographic separation, a Kinetex (biphenyl, 50 × 2.1 mm, 1.7 *μ*m, 100 Å) analytical column (Phenomenex, Aschaffenburg, Germany) protected by a HPLC guard cartridge system (C18 Security Guard, Phenomenex) was used. The analytes were detected using the Waters Quattro Micro tandem mass spectrometer equipped with an electrospray ionization interface (ESI). Data were collected and analyzed with MassLynx™ Version 4.1 software.

### 2.6. Liquid Chromatography Conditions

Gradient elution was used for chromatographic separation of the analytes with a mobile phase consisting of 0.1% formic acid in water and acetonitrile (99 : 1, v/v, water/acetonitrile). The ionic strength and pH 3.4 were kept stable by adding 10 mM ammonium acetate salt to the aqueous phase. The amount of acetonitrile was increased after 1.0 min in the mobile phase (75 : 25, v/v, water/acetonitrile). After separation, the column was reequilibrated with starting conditions for 7 min. The chromatographic time was 10 min in total. In contrast to the original method [17], a different column was used with a smaller particle diameter as outlined above. Due to the smaller particle diameter, the flow had to be adjusted. To obtain a lower backpressure, the chromatographic influencing factor of the mobile phase flow was changed from 500 to 300 *μ*L/min as well. With a column temperature of +24°C, the retention time for hydromorphone and hydromorphone-D3 was 3.71 min.

### 2.7. Electrospray Ionization-Mass Spectrometry

Electrospray ionization-mass spectrometry (ESI-MS) was accomplished in a positive electrospray mode with multiple reaction monitoring (MRM). Nitrogen was used as the desolvation cone gas, and argon was used as the collision gas. The ion source temperature was set at 140°C. The capillary and cone voltages were 3.5 kV and 40 V, respectively, and the cone gas flow was set at 50 L/min. The drying gas temperature was 500°C, and the flow was set to 900 L/min. The product ions monitored with MRM were 286⟶185 *m*/*z* for hydromorphone and 289⟶185 *m*/*z* for the internal standard hydromorphone-D3. The dwell time was 400 ms for all ion transitions monitored.

### 2.8. Method Validation

Linearity, precision, and accuracy of the applied method were assessed according to the Food and Drug Administration (FDA) guidelines [10]. Linearity of the method was assessed using seven freshly prepared plasma calibration samples over the concentration range of 0.3–20 ng/mL. The calibration curve was determined with Targetlynx software Version 4.1 (Waters) using the least square method. Inter- and intraassay errors were assessed from QC samples prepared at low (0.313 ng/mL), middle (2.50 ng/mL), and high concentrations (20.0 ng/mL), respectively. Interassay accuracy and precision were evaluated by the analysis of five replicates of the QC samples in at least three runs within three consecutive days. For intra-assay analysis, five samples of the three different concentrations were analyzed within one day. Precision was expressed as percentage standard deviation: %RSD = 100 *∗* (SD/mean). Accuracy was expressed as percentage deviation of the measured concentration (C_measured_) from the nominal concentration (C_nominal_): %RE = 100 *∗* (C_measured_ − C_nominal_)/C_nominal_. Precision and accuracy were considered acceptable if the %RSD was less than 15%, for LLOQ less than 20% and if the %RE was within ±15%. The extraction recovery for hydromorphone and the internal standard was calculated in the first study corresponding to 100% extraction recovery.

### 2.9. Assessment of Long-Term Stability

The long-term stability of hydromorphone plasma concentrations was assessed by comparing the concentrations determined in the year 2016 (C_2016_) using the original method [17] and the concentrations determined from the thawed samples in the year 2019 using a slightly modified and enhanced method (C_2019_). The absolute concentration difference (C_2019_ − C_2016_) and the percentage deviation %RE = 100 *∗* (C_2019_ − C_2016_)/C_2016_ were determined for each sample. Summary statistics were determined within each patient and for the complete data set.

## 3. Results and Discussion

### 3.1. Chromatography and Mass Spectrometry

A low acid concentration and a high percentage of organic modifiers in the mobile phase achieved the best chromatographic separation. During separation, the fraction of acetonitrile was increased to 25%. A flow of 300 *μ*L/min could be applied without loss in the separation quality. In order to achieve a high intensity of [M + H]^+^ ions of the analytes, the conditions for mass spectrometry were tested. The positive ESI mode yielded a high abundance of fragment ions. No interference from endogenous substances in the blank plasma lots or from other metabolites was found in the retention time of hydromorphone. Chromatograms of a blank sample (blank plasma plus internal standard), a control sample (blank plasma plus standard plus internal standard), and a patient sample (patient plasma plus internal standard) are presented in Figures 1–3, respectively. This demonstrates that hydromorphone concentration in human plasma could be measured with a stable UPLC-like system and tandem mass spectrometry with multiple reaction monitoring of the daughter signals. Only few influencing factors were to be optimized to get a better signal of the analytes.

### 3.2. Linearity, Limits of Detection, and Quantification

A linear calibration curve was identified for the hydromorphone concentration within the range from 0.3 to 20 ng/mL (*y* = 918.99*x* + 448.32, *r*^2^ = 0.9989, Figure 4). The limit of detection (LOD) was 0.001 ng/mL with a signal-to-noise ratio of 13.65. The lower limit of quantification (LOQ) was 0.3 ng/mL.

### 3.3. Precision and Accuracy

The results of the modified method concerning the inter- and intra-assay precision and accuracy are summarized in Tables 1 and 2. The precision and accuracy were very good for the middle and high concentrations (%RSD<6%, %RE within ±2%) and acceptable for the low concentration at the LOQ (%RSD<15%, %RE within ±15%).

### 3.4. Long-Term Stability

Overall, 44 samples of three patients were reanalyzed to assess the stability of hydromorphone after three years. The maximum and minimum hydromorphone plasma concentrations were 0.30 and 15.3 ng/mL, respectively. Chromatograms of hydromorphone and hydromorphone-D3 from one sample (patient #36, sample #6) measured in 2016 and measured in 2019 are shown in Figure 5. High peaks for hydromorphone and hydromorphone-D3 were detected in both measurements, and the determined hydromorphone concentrations of this sample were 10.11 ng/mL and 10.98 ng/mL, respectively, with a percentage deviation of 8.6%. The results for the long-term stability are summarized in Table 3. Overall, the hydromorphone plasma concentrations determined in 2019 were 1.07% ± 14.8% lower than those determined in 2016. There was no correlation between the percentage deviation and the plasma concentration (*r*^2^ = 0.001). Therefore, one can conclude that hydromorphone concentration was stable when human plasma was frozen and stored at −20°C over a period of at least three years. One limitation of this study might be the relatively small number of analyzed blood samples. On the other hand, the samples covered a relatively large and clinically relevant concentration range of 0.3–15 ng/mL.

## 4. Conclusion

We investigated the stability of hydromorphone solved in frozen human plasma under laboratory storage conditions for a period of three years. By applying a modified and enhanced LC-MS/MS method, we could demonstrate that hydromorphone can be measured with reproducible results. This finding is of value for re-evaluations or delayed analyses in pharmacokinetic studies, but also, e.g., in forensic medicine, in cases where the samples were not initially screened for hydromorphone.

## Figures and Tables

**Figure 1:** Chromatogram of a blank sample (blank plasma plus internal standard). The internal standard hydromorphone-D3 is presented in the upper panel and hydromorphone in the lower panel, respectively.

**Figure 2:** Chromatogram of a control sample (blank plasma plus standard plus internal standard) with a concentration of 2.5 ng/mL. The internal standard hydromorphone-D3 is presented in the upper panel and hydromorphone in the lower panel, respectively.

**Figure 3:** Chromatogram of a patient sample (patient plasma plus internal standard). The internal standard hydromorphone-D3 is presented in the upper panel and hydromorphone in the lower panel, respectively.

**Figure 4:** Calibration data of hydromorphone and hydromorphone-D3 used as the internal standard for the range of 0.3 to 20 ng/mL. The black circles represent the calibration samples, and the red line represents the calibration curve determined by linear regression. The response was calculated from the area under the curve of the hydromorphone peak (AUC_HM_), the area under the curve of the internal standard peak (AUC_IS_), and the concentration of the internal standard (C_IS_): response = AUC_HM_/AUC_IS_ *∗* C_IS_.

**Figure 5:** Chromatograms of a patient sample measured in 2016 (two upper panels) and 2019 (two lower panels). The signal of hydromorphone is shown in the top panel each and the signal of internal standard hydromorphone-D3 is shown in the bottom panel each, respectively.

**Table 1:** Interassay accuracy and precision of the applied analytical method.

QC sample	Nominal concentration (ng/mL)	Mean ± SD (ng/mL)	%RSD	%RE	*n*
High concentration	20.0	19.98 ± 0.33	1.63	−0.10	15
Middle concentration	2.50	2.49 ± 0.14	5.45	−0.53	15
Low concentration	0.31	0.35 ± 0.052	14.9	10.9	15

SD: standard deviation; %RSD: relative standard deviation; %RE: relative error from nominal concentration.

**Table 2:** Intra-assay accuracy and precision of the applied analytical method.

QC sample	Nominal concentration (ng/mL)	Mean ± SD (ng/mL)	%RSD	%RE	*n*
High concentration	20.0	19.8 ± 0.47	2.35	−0.90	5
Middle concentration	2.50	2.54 ± 0.055	2.16	1.60	5
Low concentration	0.31	0.32 ± 0.045	14.0	2.40	5

SD: standard deviation; %RSD: relative standard deviation; %RE: relative error from nominal concentration.

**Table 3:** Deviation between the hydromorphone plasma concentrations when re-analyzed in 2019 from thawed samples after more than three years and the first measurements in 2016.

Patient number	Concentration difference (ng/mL)	%RE	*n*
36	−0.20 ± 0.80	−2.88 ± 13.6	15
39	0.41 ± 0.94	8.35 ± 12.7	14
43	−0.53 ± 0.76	−8.07 ± 13.7	15
Overall	−0.12 ± 0.90	−1.07 ± 14.8	44

%RE: relative deviation.

## Data Availability

The data supporting the results of this study are available from the corresponding author upon request.
